This article has been retracted.

# Interferon characterization associates with asthma and is a potential biomarker of predictive diagnosis

**DOI:** 10.1042/BSR20204210

**Published:** 2021-03-19

**Authors:** Hairong Shu, Yong Li, Hangyu Xu, Qing Yin, Jianxin Song, Minqiao Zheng, He Li

**Affiliations:** 1 Department of Otolaryngology, Taizhou Central Hospital (Taizhou University Hospital), Taizhou, Zhejiang 318000, China; 2 Department of Otolaryngology, Taizhou Municipal Hospital, Medical College of Taizhou University, Taizhou, Zhejiang 318000, China; 3 Central Laboratory, The Affiliated Wenling Hospital, Wenzhou Medical University; #333, S Chuan’an Road, Wenling, Zhejiang 317500, China; 4 Department of Otolaryngology, The First Affiliated Hospital of Wenzhou Medical University, Village ShangCai, Ouhai District, Wenzhou City, Zhejiang Province 325000, China

**Keywords:** asthma, biomarker, blood, diagnosis, IFN

## Abstract

Interferon (IFN) plays a role in immune and inflammation responses. However, the effect of IFN in asthma is still not fully clear. The present study was conducted to better understand the role of IFN signatures in asthma. Blood samples from case–control studies (study 1: 348 asthmas and 39 normal controls and validation study 2: 411 asthmas and 87 normal controls) were enrolled. The single-sample gene set enrichment analysis (ssGSEA) method was used to quantify the levels of 74 IFN signatures. Gene Ontology analysis and pathway function analysis were performed for functional analysis and a protein–protein interaction (PPI) network was constructed. The area under the curve (AUC) value was used to evaluate the diagnostic ability. In our work, IFN-γ response-DN, negative regulation of IFN-γ secretion, IFNG pathway, negative regulation of response to IFN-γ, and type 1 IFN biosynthetic process showed higher levels in asthma. Functional analysis demonstrated that pathway and biological process involved in IFN signaling pathway, regulation of type 1 IFN production and response to IFN-γ. Hub IFN-related genes were identified, and their combination as biomarker exhibited a good diagnostic capacity for asthma (AUC = 0.832). These findings offered more insight into the underlying mechanism of how IFN signatures affected asthma. The use of the easy-to-apply IFN-related genes might serve as a promising blood-based biomarker for early diagnosis of asthma.

## Introduction

Asthma, a major global public health issue, is a frequent chronic respiratory disease. This disease is characterized by variable and recurring airflow obstruction, airway inflammation, and bronchial hyperresponsiveness [1,2]. Asthma affects approximately 4.3% of the global population resulting in an increased burden on families and healthcare systems. The prevalence of asthma is increasing [3,4]. Asthma is considered as a multifactorial and heterogeneous disorder that is mainly influenced by genetic and environmental risk factors [5,6]. However, the exact and underlying mechanisms of asthma are still largely uncertain. In addition, it is not always easily diagnosed [7]. Therefore, it is necessary to further explore the potential mechanisms and find useful biomarkers of diagnosis for asthma.

The recognition that asthma is primarily associated with IgE production-related T helper type 2 (Th2) and recruitment of mast cells and eosinophils [8]. In recent years, studies suggest that T helper type 1 (Th1) cytokines are responsible for the pathogenesis of asthma. Th1 responses result in the production of interferon (IFN)-γ [9,10]. Toll-like receptor 9 (TLR9) activation is involved in AHR and airway inflammation. IFN-γ is essential for TLR9-driven suppression in asthma [11]. IFN signaling has a role in the regulation of peripheral T-cell functions [12]. IFN stimulates the expression of the endoplasmic reticulum stress-related genes and inflammation and may serve a new target for the treatment of asthma [13]. However, the role and underlying molecular regulatory of IFN signature remain largely unclear in asthma.

This comprehensive study was first conducted to determine the role of 74 IFN signatures in blood specimens of patients with asthma. In addition, we also explored IFN-related hub genes and their biological mechanisms, and we explored whether IFN could be a novel and useful biomarker in diagnosing asthma. This work could provide a more effective treatment approach and diagnostic test for asthma.

## Materials and methods

### Study 1

Expression profiling data from the microarray datasets for asthma and full-disease annotation were performed from Gene Expression Omnibus. The corresponding expression datasets with >50 participants in blood samples were included in the present work. In addition, obese asthma subjects were removed from further evaluation. Non-obese healthy subjects were used as a control group. Whole blood samples for microarray data from Affymetrix, we obtained GSE110551 and GSE137394 datasets. They were performed from the same platform GPL570 [HG-U133_Plus_2] Affymetrix Human Genome U133 Plus 2.0 Array. A robust multiarray averaging (RMA) method was adopted to normalize and process data. Moreover, the expression levels of all available genes were carried out by the log2 transformation for the quantification scale. When a gene symbol was mapped to multiple probes, the expression values of those probe sets were averaged. We integrated these two datasets to improve credibility and increase sample sizes because they were from the same platform and normalized method. Batch effects from these two datasets were corrected using the ‘ComBat’ algorithm of the ‘sva’ package [1,14]. Finally, we identified 348 cases with asthma and 39 healthy control subjects, which was considered as study 1 (discovery cohort).

### Study 2

Among a very large study population (*n*=498), we collected the expression data GSE69683 using blood samples. This dataset was from the GPL13158 platform [HT_HG-U133_Plus_PM] Affymetrix HT HG-U133+ PM Array Plate. No obese participants were observed in this study cohort. This expression dataset from asthma patients and healthy control population was normalized and processed using the RMA method. Then, we underwent the log2 transformation for data. When multiple probes mapped to the same gene, we used the mean value of those probe sets for the corresponding gene. Eventually, a total of 411 cases with asthma and 87 healthy control subjects were identified in study 2 (validation cohort).

### The levels of IFN

IFN-related signatures were collected from The Molecular Signatures Database (https://www.gsea-msigdb.org/gsea/msigdb/index.jsp). We obtained 74 IFN signatures such as IFN signaling, IFN-ɣ pathway, IFN-α response, IFN-γ response, IFN-β response, production of type I IFN, IRF3-mediated activation of type I IFN, IFN-ϒ and IFN-β secretion etc. (Supplementary Table S1). To quantify the levels of IFN signatures, we used the single-sample gene set enrichment analysis (ssGSEA) method [15,16]. The enrichment levels calculated by ssGSEA method were applied to represent the relative abundance of each IFN in each sample.

### Differentially expressed IFN genes and protein–protein interaction network

IFN-related genes were summarized from IFN signatures (Supplementary Table S2). To identify differentially expressed IFN-related genes, we performed the Wilcoxon’s test between the asthma group and the normal control group. The criteria for determining significant genes were set as adjusted *P*-value <0.05. Metascape (http://metascape.org/) is an effective tool to provide a systematic analysis resource for functional enrichment, interactome analysis, gene annotation, and membership search [17]. We uploaded significant IFN-related genes as the enrichment background for pathway analysis and biological process enrichment analysis. The enrichment terms with a *P*-value <0.01 was used as statistical significance. In addition, the protein–protein interaction (PPI) analysis was also carried out from Metascape. The network consisted of the subset of proteins that formed the interactive correlation with at least one other member. If this network included between 3 and 500 proteins, we utilized the Molecular Complex Detection (MCODE) algorithm [17,18] to identify densely connected networks and obtain the best-scoring components. According to the degree of connectivity, the PPI network identified hub genes. The PPI network was also visualized and modified using the Cytoscape software.

### Statistical analysis

To conduct difference comparisons of IFN signatures and IFN-related genes between asthma and normal control groups, Wilcoxon’s signed-rank test was applied. Receiver operating characteristic (ROC) curve is a common tool used to evaluate the discrimination accuracy of a diagnostic test [19], ROC analyses of hub genes were plotted in the current work. The area under the curve (AUC) values were quantified to determine the diagnostic accuracy to distinguish asthma and healthy control subjects using the pROC R package. All statistical *P*-values were two-sided, *P*<0.05 was considered statistically significant. All data processing was performed using R software (version: 3.5.3; R Foundation for Statistical Computing, Vienna, Austria).

## Results

### IFN signatures in asthma

Blood samples were available for 348 asthma cases and 39 non-asthma healthy controls in study 1, which was used as the discovery set. Similarly, blood samples with larger study participants from 411 asthmas and 87 healthy control subjects in study 2, which was applied for validation. We first summarized and evaluated 74 components of IFN signatures in asthma. Data from the discovery data demonstrated that a higher proportion of IFN-γ response-DN, IFN-β biosynthetic process, regulation of IFNA signaling, negative regulation of IFN-γ secretion, IFNG pathway, response to IFNG-DN, negative regulation of response to IFN-γ, type 1 IFN biosynthetic process, and positive regulation of IFNα production etc. was observed in asthma group than in healthy control group (all *P*-values <0.05) (Figure 1). We further validated these results in study 2 and found that five of these IFN signatures such as IFN-γ response-DN, negative regulation of IFN-γ secretion, IFNG pathway, negative regulation of response to IFN-γ and type 1 IFN biosynthetic process were consistent and significantly higher in asthma (all *P*-values <0.05) (Figure 2).

**Figure 1:** IFN signatures in asthma and control groups in study 1 (**A**) IFNG pathway; (**B**) IFN-γ response-DN; (**C**) IFN-β biosynthetic process; (**D**) negative regulation of IFN-γ secretion; (**E**) negative regulation of response to IFN-γ; (**F**) positive regulation of IFNα production; (**G**) type 1 IFN biosynthetic process; (**H**) LRR FLII interacting protein-1 LRRFIP1 activates type I IFN production; (**I**) regulation of IFNA signaling; (**J**) response to IFNG-DN.

**Figure 2:** IFN signatures in asthma and control groups in study 2 (**A**) IFNG pathway; (**B**) IFN-γ response-DN; (**C**) negative regulation of IFN-γ secretion; (**D**) negative regulation of response to IFN-γ; (**E**) type 1 IFN biosynthetic process.

### Differentially expressed IFN-related genes and function analysis

Using the Wilcoxon’s test, IFN-related genes from IFN signatures were analyzed in asthma and normal control groups. Finally, 322 significant genes with an adjusted *P*-value <0.05 were found in the study. We further performed a functional analysis for significant genes using Metascape. We confirmed that pathway and biological process analyses were mainly involved in regulation of innate immune response, IFN signaling pathway, regulation of type 1 IFN production and response to IFN-γ (Figure 3A).

**Figure 3:** Functional analysis and the PPI network (**A**) GO and pathway enrichment analysis; (**B**) the hub genes from the densest PPI network.

### Hub IFN-related genes from PPI networks

The PPI network contained the interactions with at least one other member for genes. According to the MCODE algorithm, we selected the densest network and demonstrated that the hub genes (Figure 3B), such as CDK1, TUBB, RFC2, HSP90AB1, HSPA9, UBA52, GCH1, NUP85, PPP2CA, XRCC6, MAP3K1, EIF4E2, KPNA5, SEH1L, RANBP2, NUP98, NUP107, NUP214, GAPDH, NUP188, and NUP93.

### Expression of hub IFN-related genes and diagnostic capacity

Figures 4 and 5 showed the expression level of the above 21 IFN-related genes. The results demonstrated that GCH1, HSP90AB1, HSPA9, KPNA5, NUP85, NUP93, NUP107, NUP188, RANBP2, SEH1L, TUBB, UBA52, and XRCC6 had lower expression levels in asthma, the remaining eight genes CDK1, EIF4E2, GAPDH, MAP3K1, NUP98, NUP214, PPP2CA, and RFC2 had higher expression levels in asthma. Additionally, we conducted ROC curve analyses to estimate the capability of these IFN-related genes for distinguishing between asthma and control blood samples. AUC values with >0.5 for these IFN-related genes were observed, and the combination of them showed the highest AUC value with 0.832 (Figure 6). Moreover, we used brochoalveolar lavage data (GSE67940: 73 asthmas and 31 normal controls) and further observed that the combination of them also had the highest AUC value (AUC = 0.864) (Supplementary Figure S1A). These suggested that a pooled biomarker could improve the predictive accuracy for diagnosis in asthma.

**Figure 4:** Expression of 13 hub IFN-related genes showing lower in asthma than healthy control group in blood samples

**Figure 5:** Expression of eight hub IFN-related genes showing higher in asthma than healthy control group in blood samples

**Figure 6:** ROC curves of IFN-related genes and their combination to estimate their diagnostic capability in distinguishing asthma and healthy control groups

## Discussion

In the world, asthma affects a large population (>300 million). Although the treatment and management strategies have some advancements, this disease has no cure. The rate of death of this disease remains a crucial global challenge [7]. The precision medicine strategy for the diagnosis and management of asthma is still necessary [20]. Evidence suggests that Th2 cytokines are involved in the pathogenesis of asthma, currently, IL-5 and IL-4 antagonists also show promising efficacy. When considering TLR9 in asthmatic treatment, Th1 pathway activation indirectly/directly balances the overactivation of the Th2 pathway [21–23]. IFN therapy represents a new opportunity and an appropriate approach to treat asthma [13]. The role of IFN signaling is investigated in inflammation and asthma [12,13]. However, the effect of IFN signaling in asthma is still not largely known. In the current work, we carried out a comprehensive analysis to explore the pattern of IFN signatures and their potential biological mechanisms in asthma.

In our study, we first explored the role of 74 IFN signatures in blood specimens of patients with asthma and observed that five IFN signatures (IFN-γ response-DN, negative regulation of IFN-γ secretion, IFNG pathway, negative regulation of response to IFN-γ, and type 1 IFN biosynthetic process) exhibited a higher level in asthma group than in healthy control group. In addition, the analysis of biological processes and pathways was still involved in regulation of type 1 IFN production, response to IFN-γ, and IFN signaling pathway. Based on the MCODE algorithm, 21 hub IFN-related genes were observed in this work. In a large population-based case–control study (411 patients with asthma and 87 healthy control subjects), these 21 IFN-related genes were performed to evaluate whether their combination can improve diagnostic ability for asthma, which suggested a more effective blood-based biomarker for diagnosing asthma in clinic.

Numerous studies have suggested that the ssGSEA method can represent the relative abundance of gene set signature and explore the underlying molecular mechanism in tumor [24–26]. In the airway epithelium, IFN-λ plays key roles in the mucosal immune response to viral infection for asthma [27]. The expression of IFN‐β and IFN‐λ1/IL‐29 was higher in asthmas compared with healthy subjects [28]. In the current work, we first determined 74 IFN signatures in asthma. IFN-γ response-DN, negative regulation of IFN-γ secretion, IFNG pathway, negative regulation of response to IFN-γ, and type 1 IFN biosynthetic process displayed higher proportion in blood samples of asthma. Using brochoalveolar lavage data (GSE67940), we further found that some IFN signatures (i.e., IFN-γ response-DN) were also higher in asthma (Supplementary Figure S1). These findings suggested that some IFN signatures had pivotal roles in the pathogenesis of asthma. Asthma is an uncontrolled disease, with a substantial mortality and morbidity burden. Because under- and overdiagnosis and misdiagnosis are common in clinical practice for asthma, thus, asthma shows a large challenge for the diagnosis and management [7]. Here, we identified 21 hub IFN-related genes and pooled these genes in blood samples of asthma. We found that asthmatic subjects exhibited a superior AUC value of the combination of biomarkers compared with control subjects (AUC = 0.832). Because of the easy‐to‐use whole blood samples, our work revealed the use of IFN-related gene biomarkers can be regarded as a useful tool for early detection and intervention of asthma.

The present study had several limitations. First, our work was a retrospective design. Second, because of insufficient data on different groups (such as allergic asthma and non-allergic asthma and exacerbated asthma condition), we did not perform the relevant analysis for different types of asthmatic groups. Finally, the survival data were not available for asthma, additional studies are necessary to validate the correlation between the survival data and asthma for the selected IFN genes in the future.

In conclusion, we identified that some IFN signatures were associated with asthma. Based on the use of blood samples, the combination of IFN-related genes demonstrated a robust and effective diagnostic ability for early detection of asthma. These findings offered the first evidence to better understand the underlying molecular mechanisms of how IFN pathways signatures affected asthma. However, further research is still necessary to elucidate the role of IFN signatures in asthma in the future.

## Supplementary Material

Supplementary Figure S1

Supplementary Tables S1-S2

## Data Availability

All data were available in this manuscript.

## Abbreviations

AHR: airway hyperreactivity
AUC: area under the curve
DN: down
IFN: interferon
IFNG: interferon gamma
IgE: immunoglobulin E
IL-4/5: interleukin-4/5
IL-29: interleukin-29
IRF3: interferon regulatory factor 3
MCODE: Molecular Complex Detection
PPI: protein–protein interaction
RMA: robust multiarray averaging
ROC: receiver operating characteristic
ssGSEA: single-sample gene set enrichment analysis
Th1/2: T helper type 1/2
TLR9: Toll-like receptor 9

## References

[1] Wu X., Wang P., Zhang Y., Gao L., Zheng B., Xu Y.et al. (2020) Toll-like receptor characterization correlates with asthma and is predictive of diagnosis. DNA Cell Biol. 39, 1313–1321 10.1089/dna.2020.554332543891

[2] Singh S.R., Sutcliffe A., Kaur D., Gupta S., Desai D., Saunders R.et al. (2014) CCL2 release by airway smooth muscle is increased in asthma and promotes fibrocyte migration. Allergy 69, 1189–1197 10.1111/all.1244424931417PMC4215601

[3] Khan I., Ul-Haq Z., Shaheen A., Zaman M., Ahmad N., Abbasi R.et al. (2018) Association of arg16gly and gln27glu, b2-adrenergic receptor gene polymorphism with asthma. A systematic review and meta-analysis of case control studies. J. Pak. Med. Assoc. 68, 90–97 29371726

[4] Loftus P.A. and Wise S.K. (2016) Epidemiology of asthma. Curr. Opin. Otolaryngol. Head Neck Surg. 24, 245–249 10.1097/MOO.000000000000026226977741

[5] Machluf Y., Farkash R., Rotkopf R., Fink D. and Chaiter Y. (2020) Asthma phenotypes and associated comorbidities in a large cohort of adolescents in Israel. J. Asthma 57, 722–735 10.1080/02770903.2019.160474331017024

[6] Toskala E. and Kennedy D.W. (2015) Asthma risk factors. Int. Forum Allergy Rhinol. 5, S11–S16 10.1002/alr.2155726335830PMC7159773

[7] Gruffydd-Jones K. (2019) Unmet needs in asthma. Ther. Clin. Risk Manag. 15, 409–421 10.2147/TCRM.S16032730936704PMC6422410

[8] Holgate S.T. (2012) Innate and adaptive immune responses in asthma. Nat. Med. 18, 673–683 10.1038/nm.273122561831

[9] Tumes D.J., Papadopoulos M., Endo Y., Onodera A., Hirahara K. and Nakayama T. (2017) Epigenetic regulation of T-helper cell differentiation, memory, and plasticity in allergic asthma. Immunol. Rev. 278, 8–19 10.1111/imr.1256028658556

[10] Wohlleben G. and Erb K.J. (2006) Immune stimulatory strategies for the prevention and treatment of asthma. Curr. Pharm. Des. 12, 3281–3292 10.2174/13816120677819411417020534

[11] Thio C.L., Lai A.C., Chi P.Y., Webster G. and Chang Y.J. (2019) Toll-like receptor 9-dependent interferon production prevents group 2 innate lymphoid cell-driven airway hyperreactivity. J. Allergy Clin. Immunol. 144, 682e9–697e9 10.1016/j.jaci.2019.03.00830914379

[12] Gonzales-van Horn S.R. and Farrar J.D. (2015) Interferon at the crossroads of allergy and viral infections. J. Leukoc. Biol. 98, 185–194 10.1189/jlb.3RU0315-099R26026068PMC4501675

[13] Bhakta N.R., Christenson S.A., Nerella S., Solberg O.D., Nguyen C.P., Choy D.F.et al. (2018) IFN-stimulated gene expression, type 2 inflammation, and endoplasmic reticulum stress in asthma. Am. J. Respir. Crit. Care Med. 197, 313–324 10.1164/rccm.201706-1070OC29064281PMC5811952

[14] Leek J.T., Johnson W.E., Parker H.S., Jaffe A.E. and Storey J.D. (2012) The sva package for removing batch effects and other unwanted variation in high-throughput experiments. Bioinformatics 28, 882–883 10.1093/bioinformatics/bts03422257669PMC3307112

[15] Yi M., Nissley D.V., McCormick F. and Stephens R.M. (2020) ssGSEA score-based Ras dependency indexes derived from gene expression data reveal potential Ras addiction mechanisms with possible clinical implications. Sci. Rep. 10, 10258 10.1038/s41598-020-66986-832581224PMC7314760

[16] Bindea G., Mlecnik B., Tosolini M., Kirilovsky A., Waldner M., Obenauf A.C.et al. (2013) Spatiotemporal dynamics of intratumoral immune cells reveal the immune landscape in human cancer. Immunity 39, 782–795 10.1016/j.immuni.2013.10.00324138885

[17] Zhou Y., Zhou B., Pache L., Chang M., Khodabakhshi A.H., Tanaseichuk O.et al. (2019) Metascape provides a biologist-oriented resource for the analysis of systems-level datasets. Nat. Commun. 10, 1523 10.1038/s41467-019-09234-630944313PMC6447622

[18] Bader G.D. and Hogue C.W. (2003) An automated method for finding molecular complexes in large protein interaction networks. BMC Bioinformatics 4, 2 10.1186/1471-2105-4-212525261PMC149346

[19] Obuchowski N.A. and Bullen J.A. (2018) Receiver operating characteristic (ROC) curves: review of methods with applications in diagnostic medicine. Phys. Med. Biol. 63, 07TR1 10.1088/1361-6560/aab4b129512515

[20] Canonica G.W., Ferrando M., Baiardini I., Puggioni F., Racca F., Passalacqua G.et al. (2018) Asthma: personalized and precision medicine. Curr. Opin. Allergy Clin. Immunol. 18, 51–58 10.1097/ACI.000000000000041629189350

[21] Peters M.C. and Wenzel S.E. (2020) Intersection of biology and therapeutics: type 2 targeted therapeutics for adult asthma. Lancet 395, 371–383 10.1016/S0140-6736(19)33005-332007172PMC8522504

[22] Katsaounou P., Buhl R., Brusselle G., Pfister P., Martinez R., Wahn U.et al. (2019) Omalizumab as alternative to chronic use of oral corticosteroids in severe asthma. Respir. Med. 150, 51–62 10.1016/j.rmed.2019.02.00330961951

[23] Long A.A. (2009) Monoclonal antibodies and other biologic agents in the treatment of asthma. MAbs 1, 237–246 10.4161/mabs.1.3.835220065638PMC2726591

[24] Berger A.C., Korkut A., Kanchi R.S., Hegde A.M., Lenoir W., Liu W.et al. (2018) A comprehensive pan-cancer molecular study of gynecologic and breast cancers. Cancer Cell 33, 690.e9–705.e9 10.1016/j.ccell.2018.03.01429622464PMC5959730

[25] Verhaak R.G., Tamayo P., Yang J.Y., Hubbard D., Zhang H., Creighton C.J.et al. (2013) Prognostically relevant gene signatures of high-grade serous ovarian carcinoma. J. Clin. Invest. 123, 517–525 2325736210.1172/JCI65833PMC3533304

[26] Zhang B., Wu Q., Li B., Wang D., Wang L. and Zhou Y.L. (2020) m(6)A regulator-mediated methylation modification patterns and tumor microenvironment infiltration characterization in gastric cancer. Mol. Cancer 19, 53 10.1186/s12943-020-01170-032164750PMC7066851

[27] Niwa M., Fujisawa T., Mori K., Yamanaka K., Yasui H., Suzuki Y.et al. (2018) IL-17A attenuates IFN-lambda expression by inducing suppressor of cytokine signaling expression in airway epithelium. J. Immunol. 201, 2392–2402 10.4049/jimmunol.180014730224514

[28] da Silva J., Hilzendeger C., Moermans C., Schleich F., Henket M., Kebadze T.et al. (2017) Raised interferon-beta, type 3 interferon and interferon-stimulated genes - evidence of innate immune activation in neutrophilic asthma. Clin. Exp. Allergy 47, 313–323 10.1111/cea.1280927622317

